The article "Comparison between Percutaneous Kyphoplasty and Posterior Fixation Combined with Vertebroplasty in the Treatment of Stage III Kümmell's Disease without Neurological Deficit" was published in 2022. Journal: Biomed Res Int.

# Comparison between Percutaneous Kyphoplasty and Posterior Fixation Combined with Vertebroplasty in the Treatment of Stage III Kümmell's Disease without Neurological Deficit

**DOI:** 10.1155/2022/2193895

**Published:** 2022-09-08

**Authors:** Yijie Liu, Yi Zhu, Renjie Li, Weimin Jiang, Huilin Yang

**Affiliations:** ^1^Department of Orthopaedic Surgery, The First Affiliated Hospital of Soochow University, 899 Pinghai Street, Suzhou 215006, China; ^2^Department of Orthopaedic Surgery, Dushu Lake Hospital Affiliated to Soochow University, 9 Chongwen Road, Suzhou, Jiangsu Province 215124, China

## Abstract

**Objective:**

To evaluate the clinical and radiological outcomes of percutaneous kyphoplasty (PKP) versus posterior fixation combined with vertebroplasty PF+VP for treating stage III Kümmell's disease (KD) patients without neurological deficits.

**Methods:**

From April 2016 to February 2020, a total of 88 patients with single-level stage III KD without neurological deficits, including 45 patients treated by PKP and 43 patients who underwent posterior fixation combined with vertebroplasty PF+VP, were retrospectively studied. The outcome parameters, including blood loss, operative time, kyphotic Cobb angle, height of vertebrae, Oswestry Disability Index (ODI), and visual analog scale (VAS) score, were compared between the PKP group and the PF+VP group.

**Results:**

The mean follow-up time was 29.3 ± 7.0 months, ranging from 24 to 48 months. The kyphotic angle and vertebral height in both groups were significantly improved compared with those before surgery at three days, 3 months and the final follow-up. The estimated blood loss, operative time, and length of stay were significantly lower in the PKP group than in the PF+VP group (*P* < 0.001). The FP+VP group showed better results in kyphotic angle correction than the PKP group (*P* = 0.024). In the short-term follow-up (up to 3 months), the PKP group had lower VAS and ODI scores than the PF+VP group. In contrast, there were no significant differences between the two groups (*P* > 0.05) at the final follow-up. The average cost of PKP was lower than that of PF+VP.

**Conclusion:**

The results of our study showed that both PKP and PF+VP were safe and effective for stage III KD patients without neurological deficits. Although PF+VP presents better performance in kyphotic angle correction, PKP was associated with less surgical trauma, quicker pain relief, and lower expense than PF+VP. Therefore, it can be considered an alternative option for patients with advanced KD.

## 1. Introduction

Kümmell's disease (KD) was first described by German scholar Kümmell in 1895 [1], presenting a progressive development varying from the occurrence of minor fracture to mild vertebral collapse and instability and finally to severe vertebral collapse, which would be very likely to compress the spinal cord, resulting in neurological deficits. Hence, an aggressive treatment is needed for KD.

Percutaneous kyphoplasty (PKP) can strengthen the vertebral body and relieve pain instantly; it has been widely applied in recent years and has achieved satisfactory clinical results in stage I or II KD [2, 3]. There is a consensus that open surgery should be applied in stage III KD with neurological deficits. Nevertheless, the surgical option in stage III KD without neurological deficits remains controversial. Some scholars hold the view that it is difficult to perform PKP in KD due to the high risk of bone cement leakage, so they define stage III KD as a relative contraindication of PKP [4, 5]. We performed this retrospective study to compare the clinical results of PKP and PF+VP for treating stage III KD patients without neurological deficits.

## 2. Methods

### 2.1. Patients

This is a retrospective and comparative clinical study. From April 2016 to February 2020, a total of 88 patients with single-level stage III KD without neurological deficits received PKP or PF+VP. The patients were divided into two groups based on the surgical procedure they received. Forty-five patients with single-level stage III KD without neurological deficits who underwent PKP were classified into the PKP group. Forty-three patients who underwent posterior fixation combined with vertebroplasty PF+VP were classified into the PF+VP group. The study was approved by local Medical Ethics Committees (ethical code 2020179). Informed written consent was obtained from all individual participants. There were no statistically significant differences in patient age, sex, follow-up time, or operative levels between the PKP group and the PF+VP group.

The inclusion criteria included the following: (I) patients diagnosed with single level stage III KD by clinical symptoms and imaging data, (II) bone mineral density *T* score ≤ -2.5 SD, and (III) magnetic resonance imaging (MRI) manifested spinal cord compression, but no symptomatic neurological deficit existed. The exclusion criteria included (I) bilateral pedicle comminuted fracture; (II) pathological vertebral fractures, such as spinal metastasis and tuberculosis; (III) stage III KD with neurological deficits; and (IV) patients with severe cardiopulmonary and hepatorenal dysfunction who could not tolerate the operation. All patients who met the criteria were included.

### 2.2. Operative Procedure

#### 2.2.1. Percutaneous Kyphoplasty (PKP)

After general anesthesia, the patient was placed in the prone position, with pillows under the chest and waist to maintain the hyperextension position. The injured vertebrae were confirmed by taking anteroposterior and lateral images by the C-arm. Then, bilateral transpedicular working channels were inserted by the cannula and trocar systems. After that, bilateral balloons were placed into the intravertebral vacuum cleft below the superior endplate. The balloon was carefully inflated to elevate the superior endplate, achieving height restoration and kyphosis correction. Polymethylmethacrylate (PMMA) bone cement was slowly injected to the point where balloon inflated, and the cavity was filled. All steps were performed under the guidance of the C-arm.

### 2.3. Posterior Fixation Combined with Vertebroplasty PF+VP

The procedure was performed under general anesthesia and in a prone hyperextension position with a standard midline approach. After routine exposure, 8 pedicle screws were inserted bilaterally into adjacent vertebrae, and PMMA bone cement was injected through the screw to enhance the pullout strength if necessary. Then, the 2 rods were fixed to achieve satisfactory indirect reduction. Vertebroplasty was performed for the fractured vertebra. All processes above are under the guidance of a C-arm. Autogenous bone grafts are used to facilitate posterolateral fusion. Long-segment fixation is applied instead of short-segment fixation to reduce the incidence of screw loosening, displacement, or fracture.

### 2.4. Data Collection and Outcome Assessment

All patients were routinely examined at 3 days, 1 month, 3 months, 6 months, and 12 months postoperatively and every 1 year thereafter. Clinical and radiologic data were obtained by the same physician on our team, and all operations were performed by the same surgeon.

The clinical outcomes included the Oswestry Disability Index (ODI) and visual analog scale (VAS) score. The ODI recovery rate (RR) was also calculated. RR = (preoperative ODI − postoperative ODI)/(preoperative ODI score)∗100 [6]. Estimated blood loss, operative time, and length of stay (LOS) were routinely recorded.

The anterior and central heights of the fractured vertebrae and adjacent vertebrae were measured on a lateral radiograph. The ratio of vertebral height = (height of fractured vertebrae)/(mean height of adjacent vertebrae)∗100%. The kyphotic Cobb angle was measured using Cobb's method, which is formed by the lines along the superior endplate of the upper vertebrae and the inferior endplate of the lower vertebrae in the standard lateral radiograph (Figure 1).

All analyses were performed using SPSS Statistics version 20.0 (IBM Corp, Armonk, New York). The results are presented as simple descriptive statistics (mean and standard deviation for continuous variables, frequency, and percentage for categorical variables). Preoperative and postoperative data, including ODI and VAS scores, the height of fractured vertebrae, and the kyphotic Cobb angle, were assessed using repeated-measures ANOVA. The LSD test was used for multiple comparisons. The results were considered significant when *P* < 0.05.

## 3. Results

### 3.1. Demographics and Perioperative Outcomes

All surgeries were successfully performed, and all patients were followed up for at least 24 months with a mean follow-up period of 29.3 ± 7.0 months (range: 24-48 months). Compared with the PKP group, the PF+VP group had more blood loss during the operation (16.8 ± 8.9 ml for PKP vs. 288.1 ± 89.7 ml for PF+VP, *P* < 0.001), required a longer operative time (43.8 ± 17.1 min for PKP vs. 94.4 ± 20.5 min for PF+VP, *P* < 0.001), and needed a longer LOS (5.3 ± 1.1 days for PKP vs. 7.5 ± 1.4 days for PF+VP, *P* < 0.001) (Table 1).

### 3.2. Clinical Outcomes

The mean VAS scores improved significantly from preoperative to the final follow-up, descending from preoperation (9.0 ± 0.8) to final follow-up (1.5 ± 1.0) in the PKP group and from preoperation (9.1 ± 0.7) to final follow-up (1.4 ± 1.0) in the PF+VP group. The ODI scores decreased significantly from preoperation to the last follow-up, descending from 77.0 ± 9.7 to 30.3 ± 5.4 in the PKP group and from 76.9 ± 9.9 preoperatively to 29.5 ± 4.0 postoperatively in the PF+VP group. The ODI RR at the final follow-up was 60.1% ± 9.3% and 61.2% ± 6.5% for the PKP and PF+VP groups, respectively. The difference between the 2 groups was statistically significant in VAS, ODI, and RR at 3 days and 3 months postoperatively, which was lower in the PKP group than in the PF+VP group. In contrast, there was no significant difference between the two groups at the final follow-up. The VAS, ODI, and RR data are summarized in Table 2.

### 3.3. Radiologic Outcomes

The preoperative Cobb angle showed no significant difference between the groups (29.5° ± 9.3° for PKP vs. 30.5° ± 7.7° for PF+VP, *P* > 0.05). However, the PF+VP group showed better results in kyphotic angle correction than the PKP group (19.7° ± 3.4° for PKP vs. 16.5° ± 3.3° for PF+VP, *P* = 0.024 at final follow-up). In the PKP group, the ratio of anterior vertebral height increased from preoperation (26.9 ± 6.2 mm) to postoperation (37.9 ± 5.0 mm), and the ratio of central vertebral height increased from preoperation (31.3 ± 8.5 mm) to postoperation (52.4 ± 6.1 mm) at the final follow-up. In the PF+VP group, the corresponding parameters significantly increased from preoperation (28.1 ± 7.5 mm) to postoperation (38.2 ± 5.1 mm) and from preoperation (30.7 ± 9.0 mm) to postoperation (51.9 ± 6.7 mm) at the final follow-up. The kyphotic Cobb angle and vertebral height at the final follow-up were significantly corrected when compared with the preoperative values in both groups. The radiological evaluation results are summarized in Table 3. Typical cases of both groups are shown in Figures 1–3.

### 3.4. Complications

Ten patients in the PKP group had asymptomatic cement leakage, including 6 intervertebral cases, 3 anterior-vertebral cases, and 1 paravertebral case, and the incidence of cement leakage in the PKP group was 22.2%. One case of adjacent segment fracture occurred during hospitalization, and two cases were observed at follow-up. All of them received PKP again and recovered well. In the PF+VP group, 9 patients had asymptomatic cement leakage, and the incidence of cement leakage was 20.9%. One case of another segment fracture was observed at follow-up time and received PKP treatment again. There was one case of incision infection that was restored after dressing for 10 days in the PF+VP group. There were no hemorrhages in either group, and there were no instances of bolt loosening or rupture of screws in the PF+VP group.

## 4. Discussion

KD is defined as vascular osteonecrosis of the vertebral body and usually occurs after OVCF [7, 8]. It may lead to back pain, spinal canal stenosis, or neurological deficits that reduce quality of life and increase the risk of disability or even mortality. Conservative treatments include bed rest, medical pain control, rigid back support, and antiosteoporosis drugs, all of which achieve poor effects, leading to progressive vertebral collapse and kyphotic deformities. Therefore, aggressive surgical intervention is sometimes recommended.

According to the clinical classification by Li et al. [9], KD was divided into three stages. In the first stage, the vertebral body is slightly injured by minor trauma, and the loss of vertebral height is less than 20%. In the second stage, dynamic instability of vertebral bodies leads to fracture, and the loss of vertebral height is more than 20%, but the posterior wall of the vertebral body remains intact. In the third stage, the posterior wall collapses and leads to continuous severe back pain, with or without neurological deficits. The optimal surgical option in stage III KD without neurological deficits remains unclear. Traditional surgical targets are mainly vertebral canal decompression, orthopedic bone grafts, and internal fixation, including anterior and posterior surgery. Anterior surgery can lead to thorough decompression, and reconstruction of the anterior column stability, and it will not affect the posterior column structure; however, level of surgical trauma is high, it is easy for the implant to appear to be sinking or loose, and complications may occur, ultimately affecting the surgical curative effect [5]. Posterior surgery for stage III KD, decompression, osteotomy, and multiple pedicle screw fixation are often used, resulting in large surgical trauma and large blood loss [10]. The failure rate of internal fixation is very high in both anterior and posterior approaches due to severe osteoporosis [11–13]. In addition, many elderly patients cannot tolerate open surgery. Therefore, for stage III KD without neurological deficits, open operation might not be the first choice. PKP is a minimally invasive surgery with less surgical trauma that enables patients to walk on the first day after PKP surgery and avoids a series of complications caused by a long time in bed, such as lung infection and deep vein thrombosis of both lower limbs. Additionally, PKP does not require pedicle screw fixation, only vertebral augmentation, and therefore, the surgical cost is lower than that of PF+VP.

The feasibility of PKP in the treatment of stage III KD without neurologic deficit.

Some scholars hold the view that PKP is considered to be a relative contraindication in treating advanced KD due to the difficulty of puncture, incomplete posterior vertebral body wall, and high leakage rate of bone cement [5, 14]. Nevertheless, PKP and PVP have been proven effective in treating stage I or II KD [3, 15–21]. Xia et al. examined 50 patients with KD who underwent PKP, and all of them showed significant improvement in pain, vertebral height, and kyphotic Cobb angle after 2 years of follow-up [20]. Lu et al. [21] compared PKP and short-segmental fixation combined with vertebroplasty and concluded that both methods are safe and effective for KD, while PKP can shorten the operation time and reduce the volume of blood loss. However, few studies have reported on PKP in the treatment of stage III KD. Based on the amount of clinical practice, we consider PKP feasible for treating stage III KD without neurologic symptoms. After anesthesia, the patient was placed in the hyperextension position. By tractive force from the intervertebral disc and the anterior longitudinal ligament, the vertebral height could be partially recovered, and the cleft might be enlarged. Intravertebral vacuum clefts are usually wrapped around fibrous tissue and can therefore decrease the leakage rate of bone cement. Although our results showed that PF+VP is better than PKP in kyphotic angle correction, PKP has advantages of smaller surgical trauma, quicker pain relief, lower expense, and avoidance of open surgery complications. Furthermore, if PKP fails to relieve pain, open surgery can still be performed as a remedial measure.

Our experience in PKP treating stage III KD without neurologic symptoms.

First, intravertebral vacuum cleft is the basis for the PKP technique. Even if the vertebral body is seriously collapsed, the posterior wall of the vertebral body is incomplete or the corresponding segment of the vertebral canal is compressed, and an intravertebral vacuum cleft can provide space for balloon dilatation and bone cement injection, thus enabling the use of PKP for the treatment of stage III KD. Hence, a thorough imaging examination is necessary to decide whether PKP can be performed [22, 23]. The procedure of putting pins into the cleft accurately is crucial and is the key to decreasing the incidence of leakage of bone cement.

Second, ideal position and proper dilation of the balloon are essential. Slow and moderate dilation of the balloon can not only correct kyphosis and restore the vertebral height but also provide conditions for bone cement filling under high viscosity and low pressure to reduce the leakage of bone cement. The 3/4 anterior part of the vertebra should be the ideal position of the balloon. Close to the anterior edge, the anterior fibrous capsule would be ruptured. In contrast, close to the posterior edge damages, the posterior capsule and results in pushing bone mass into the spinal canal. To prevent leakage, we concluded the following: (1) The pin must be put directly into the IVC, which is the key procedure. (2) The balloon should be placed at 3/4 of the anterior side of the vertebrae and dilated slowly and moderately. (3) Early-period bone cement should be injected in 1/3 of the anterior part and checked by C-arm every 1 ml, in addition to checking every 0.5 ml after injection in the 1/3 middle part and checking every 0.25 ml after injecting late-period cement in the 1/3 posterior part. Once leakage occurs, injection should be stopped immediately. The posterior wall can be tightened and partially reduced by the force of the posterior longitudinal ligament after a prone position. When injecting the bone cement, the injection was stopped immediately when the cement diffused to the collapsed posterior wall.

Third, the amount of bone cement is important. Excessive bone cement increases the incidence of leakage, while insufficient bone cement cannot provide enough support. According to our experience, the amount of bone cement is proper when the volume of cement is slightly larger than that of balloon dilation or the push rod has a withdrawal force during injection. For patients with anterior wall defects, a small quantity of middle-late phase bone cement should be injected first to seal the cleft before early phase bone cement injection, which promotes dispersion of cement and increases the riveting force with surrounding bone. In our study, the rate of asymptomatic cement leakage was 13.3%, which is lower than the 47.8%-91.9% reported in the previous literature [11, 24, 25].

According to our study, we found that both PKP and PF+VP techniques are safe and effective for stage III KD without neurological deficits. Although patients with a severe kyphotic angle may take PF+VP as the first choice, PKP is still an effective and less invasive method for pain relief. Blood loss and operation time were lower in the PKP group, avoiding complications of open surgery. Furthermore, ODI and VAS did show significant differences within 1 month follow-up but not at 3 months follow-up and thereafter, indicating that PKP has smaller surgical injury and quicker pain relief than PF+VP. Additionally, the medical expense of PKP is lower than that of PF+VP.

This study has several limitations. First, this study is a retrospective analysis, and no method was adopted to ensure unbiased randomization of the 2 groups. Although we did include all the patients in our hospital database during the study period and clinical as well as radiologic data were obtained by the same physician on our team and all the operations were performed by the same surgeon, the selection bias still cannot be completely eliminated. Second, patients with neurological deficits were excluded, so it is not sufficient to prove the efficacy of PKP for decompression and reestablishment of the posterior wall. In addition, the number of cases and centers were quite limited. Therefore, further large-sample and randomized controlled trials are needed.

## 5. Conclusions

The results of our study showed that both PKP and PF+VP were safe and effective for stage III KD without neurological deficits. Although PF+VP presents better performance in kyphotic angle correction, PKP was associated with less surgical trauma, quicker pain relief, and lower expense than PF+VP. Therefore, it can be considered an alternative option for patients with advanced KD.

## Figures and Tables

**Figure 1:** Images of a 77-year-old female patient. (a, b) Preoperative radiograph, manifesting the collapsed vertebra. The red line shows the Cobb angle was 11°, and the white line and the black line refers to anterior and central vertebral height, respectively. The ratio of anterior vertebral height (RAVH) was 21.4%, and the ratio of central vertebral height (RCVH) was 22.9%. (c) Preoperative CT showed the collapsed posterior wall and intravertebral cleft. (d) Preoperative MRI showed the spinal compression. (e–g) Postoperative images: the Cobb angle recovered to 8°, the RAVH was 32.5%, and the RCVH 33.4%.

**Figure 2:** Images of a 72-year-old female patient. (a) Preoperative lateral radiograph shows the Cobb angle was 24°. (b) Preoperative CT shows the intravertebral vacuum cleft exists. (c, f) Preoperative MRI and axial CT scan show the collapsed posterior wall but spinal cord compression was not quite severe. (d, e) Postoperative radiographs show the Cobb angle recovered to 16°.

**Figure 3:** Images of a 79-year-old female patient. (a–c) Preoperative images show the Cobb angle was 45°, and the vertebra was extremely compressed, but no obvious spinal cord compression. (d, e) Postoperative radiograph shows the Cobb angle recovered to 21°.

**Table 1:** Demographic and perioperative data.

	PKP group	PF+VP group	*P* value
Patients no.	45	43	
Sex			
Male	7 (15.6%)	8 (18.6%)	0.708
Female	38 (84.4%)	35 (81.4%)	
Age (years)	74.8 ± 6.4	75.8 ± 6.1	0.493
Follow-up period (months)	28.8 ± 7.4	29.8 ± 6.6	0.481
Estimated blood loss (ml)	16.8 ± 8.9	288.1 ± 89.7	<0.001
Operative time (mins)	43.8 ± 17.1	94.4 ± 20.5	<0.001
Length of stay (days)	5.3 ± 1.1	7.5 ± 1.4	<0.001

**Table 2:** Comparison of VAS, ODI, and RR.

Parameters	PKP group	PF+VP group	*P* value
VAS scores			
Preoperative	9.0 ± 0.8	9.1 ± 0.7	0.775
Postoperative 3 days	4.0 ± 1.0	6.5 ± 0.9	<0.001
Postoperative 3 months	1.8 ± 1.1	4.1 ± 0.9	<0.001
Final follow-up	1.5 ± 1.0	1.4 ± 1.0	0.742
ODI scores			
Preoperative	77.0 ± 9.7	76.9 ± 9.9	0.964
Postoperative 3 days	47.9 ± 9.6	67.3 ± 8.7	<0.001
Postoperative 3 months	31.3 ± 6.4	47.9 ± 8.2	<0.001
Final follow-up	30.3 ± 5.4	29.5 ± 4.0	0.448
RR (%)			
Postoperative 3 days	36.8 ± 13.8	11.5 ± 14.4	<0.001
Postoperative 3 months	58.4 ± 11.2	37.1 ± 11.0	<0.001
Final follow-up	60.1 ± 9.3	61.2 ± 6.5	0.508

VAS: visual analogue scale; ODI: Oswestry Disability Index. RR = (preoperative ODI − postoperative ODI)/(preoperative ODI score)∗100%.

**Table 3:** Comparison of radiological evaluation results.

Parameters	PKP group	PF+VP group	*P* value
Cobb angle (°)			
Preoperative	29.5 ± 9.3	30.5 ± 7.7	0.397
Postoperative 3 days	20.4 ± 4.3	17.2 ± 3.0	0.013
Postoperative 3 months	18.8 ± 3.9	16.7 ± 2.6	0.019
Final follow-up	19.7 ± 3.4	16.5 ± 3.3	0.024
The ratio of anterior vertebral height (%)			
Preoperative	26.9 ± 6.2	28.1 ± 7.5	0.183
Postoperative 3 days	37.6 ± 5.1	36.5 ± 4.9	0.356
Postoperative 3 months	38.1 ± 4.8	37.9 ± 5.2	0.514
Final follow-up	37.9 ± 5.0	38.2 ± 5.1	0.482
The ratio of central vertebral height (%)			
Preoperative	31.3 ± 8.5	30.7 ± 9.0	0.135
Postoperative 3 days	51.7 ± 6.6	52.5 ± 7.2	0.477
Postoperative 3 months	51.9 ± 6.4	51.3 ± 7.0	0.804
Final follow-up	52.4 ± 6.1	51.9 ± 6.7	0.539

The ratio of vertebral height = (height of fractured vertebrae)/(mean height of adjacent vertebrae)∗100%.

## Data Availability

The datasets used and/or analyzed during the current study are available from the corresponding author on reasonable request.
